The article "Risk Assessment and Regulation Algorithm for Financial Technology Platforms in Smart City" was published in 2022. Journal: Comput Intell Neurosci.

# Risk Assessment and Regulation Algorithm for Financial Technology Platforms in Smart City

**DOI:** 10.1155/2022/9903364

**Published:** 2022-03-25

**Authors:** Xiaoxi Liu, Xiaoling Yuan, Rui Zhang, Nan Ye

**Affiliations:** ^1^School of Economics and Finance, Xi'an Jiaotong University, Xi'an City 710049, Shaanxi, China; ^2^Xi'an Institute of Space Radio Technology, Xi'an City 710100, Shaanxi, China

## Abstract

The informatization of cities has been further promoted, and the construction of smart cities supported by technological innovation has been upgraded. The financial industry and data are closely related. Whether the financial industry can make good use of new information technology is the key to its successful transformation. The development of smart cities has a significant effect on the development of people's livelihood, the process of urbanization, the use of technology, the solution of urban problems, and the improvement of economic levels. This also provides a good choice for the development of cities in each country. For better development, it needs technical support. Therefore, it is very important to improve the technical level. This research mainly discusses the risk assessment and regulation algorithms of financial technology platforms in smart cities. This study divides the risk decision channels into two paths based on the smart city theory, considers the internal risk factors and external risk factors of the robo-advisory service platform from the three perspectives of platform characteristics, corporate characteristics, and investor characteristics and exploring the construction of a robo-advisory service platform risk prediction model based on the machine learning perspective. The design and implementation of a personalized financial investment prototype system, a Python-based web development framework Django, and a variety of toolkits have realized a B/S architecture robo-advisor. Among them, the function of buying and selling ETF and the trend recording function after buying are realized by simulating the transaction data collected by the data collection module. The study found that the key potential characteristics that constitute platform risks are mainly the listing year of the background company, the age of the platform, the investment threshold, and the search index. To a certain extent, this provides data support for investors and regulatory authorities to evaluate platform capabilities and platform selection. Investors should comprehensively consider platform qualifications when making platform decisions and pay attention to information such as the age of listing of companies with platform background, platform age, and investment thresholds. Only when the quality of people is improved, the quality of the population of this city improves, so that the development of the city has a broad room for growth. The accuracy of the similar formula calculation method in the big data proposed in this study reached 88%. This research provides new ideas for perfecting the black box regulatory system of robo-advisory algorithms.

## 1. Introduction

Based on the integration and utilization of resources, smart cities cooperate with terminal equipment through informatization to achieve the improvement of the level of urban governance, thereby enhancing the intelligence and technology of infrastructure. The acceleration of the network upgrade has further promoted the development of various fields. Financial information is constantly emerging, and a large amount of information can indeed help people understand the financial market more fully, but it also increases the difficulty for users to obtain effective information and reduces efficiency. Through the intelligent integration and analysis of data resources, it provides an important reference for government decision-making and has a significant role in urban governance, economic growth, and improvement of people's livelihood.

Internet finance can be regarded as the basic version of financial technology, and financial technology is its upgraded version. Compared with Internet finance, the penetration and influence of technology elements on financial technology is more obvious. Financial development can accelerate the informatization development of smart cities through technological innovation, and the efficiency of financial development plays the most prominent role. In the long run, the coordinated and orderly development of the overall financial mechanism and the close integration of technology and finance play an important role in improving the level of informatization development and accelerating the pace of smart city construction [1]. On this basis, corresponding countermeasures and suggestions are put forward to promote the integration of financial development and technological innovation to accelerate the pace of construction of smart cities in various regions.

Financial and technological developments promote each other, and financial service trade and technological advancement cherish each other. From a historical point of view, the financial service trade has emerged on the basis of trade in goods and has developed rapidly under the influence of technological progress, regulatory reforms, and economic growth. As one of the traditional industries, the financial industry is closely related to data. Whether the financial industry can make good use of new information technology is the key to its successful transformation. Menouar believes that there is no smart city without a reliable and efficient transportation system, this necessity makes ITS a key component of any smart city concept. Although traditional ITS technologies have been deployed in smart cities globally, the implementation of next-generation ITS relies on the effective integration of connected cars and autonomous vehicles, and these two technologies are undergoing extensive field testing in many cities around the world. Although these two emerging technologies are critical to the realization of fully automated transportation systems, there is still a great need for the automation of other roads and transportation components. Due to its mobility, autonomous operation, and communication/processing capabilities, UAVs are envisioned for many ITS applications. Menouar et al. described possible ITS applications that can use drones and emphasized the potential and challenges of ITS that support drones in the next generation of smart cities [2]. Bo et al. believed that data-intensive analysis is the main challenge facing smart cities due to the ubiquity of various sensors. The natural nature of geographic distribution requires new computing paradigms to provide location-aware and delay-sensitive monitoring and intelligent control. Fog computing, which extends computing to the edge of the network, fits this need. In order to protect the future community, it is necessary to integrate intelligence in the fog computing architecture, for example, perform data representation and feature extraction, identify abnormal and dangerous events, and provide the best response and control. They used an intelligent pipeline monitoring system based on fiber optic sensors and sequential learning algorithms to analyze case studies to detect events that threaten pipeline safety. A working prototype was built to experimentally evaluate the event detection performance of identifying 12 different events. These experimental results prove the feasibility of the system to be implemented in the city in the future [3]. Brundu et al. introduced an IoT software infrastructure that supports new control policies for energy management and simulated urban areas. The platform Brundu et al. proposed enables (near) real-time building energy profile interoperability and correlation with environmental data from sensors and building and grid models. In the smart city environment, the platform realizes the integration of heterogeneous data sources at the building and regional levels, and the simulation of new energy policies at the regional level. It aims to optimize energy use and consider its impact. The platform Brundu et al. proposed has been deployed in a real area, and a novel heating network control strategy has been developed and tested [4]. Mosannenzadeh believed that smart energy cities are an emerging concept in urban development, aiming to optimize the urban energy system and improve the quality of life of citizens. However, the development of smart energy cities requires a well-defined and consistent conceptual core to ensure its accurate interpretation and successful implementation. He defined the development of smart energy cities not only in the theoretical context but also in terms of practical solutions. He adopted the 5W + 1H (why, what, who, where, when, and how) model, combined with literature review and expert knowledge acquisition, namely, focus groups and interviews. This leads to (i) clarifying the general interrelationships among smart energy cities, smart cities, and sustainable cities; (ii) a holistic, multidisciplinary, and comprehensive smart energy city conceptual framework that reveals its principles, goals, intervention areas, stakeholders, and time and space scales; and (iii) a set of smart energy practical solutions and technologies, divided into eight intervention areas [5]. Badii believes that a large number of activities have been carried out in defining smart city architecture to cope with this complexity, and a large number of different types of services and processes have been implemented. He introduced the work carried out in the context of the Sii-Mobility Smart City Project. His project defines a smart city architecture that solves a wide range of processes and data. To this end, by proving the use of semantic ontology and knowledge base in data aggregation in smart service production, the latest solutions of smart city architecture based on data aggregation and smart city API are compared. Baddi's solution proposes to aggregate and re-coordinate data (open and private, static and real-time) through the use of reasoning/intelligent algorithms to achieve complex service interactions through smart city APIs. His work was developed in the context of the Sii-Mobility National Smart City Project, which combines mobility and transportation with smart city services [6]. Daniel believed that technological advancements in multiple fields have promoted the development of smart city applications, which can improve the lifestyle of modern cities. When using a visual sensor in this situation, still images and video streams can be retrieved from the monitored area, which may provide valuable data for many applications. In fact, visual sensor networks may require highly dynamic conditions to reflect changes in parameters in smart cities. In this case, the characteristics of the visual sensor and the conditions of the monitored environment, as well as the status of other concurrent monitoring systems, may affect the way the visual sensor collects, encodes, and transmits information. He proposed a fuzzy-based method to dynamically configure the operating mode of the vision sensor in sensing, encoding, and transmission modes, using different types of reference parameters. This innovative method can be considered as the basis for multisystem smart city applications based on visual surveillance, and is expected to bring significant results to this research field [7]. Smart cities ensure the sustainable economic and social development of cities by improving the efficiency of urban governance and operation. As each city faces different development foundations, the most important thing in the initial stage of smart city construction is to find a development model suitable for local characteristics. Therefore, all localities must face up to their own level of informatization development and choose a suitable road for smart city construction.

Research on the role of science and technology development in promoting cities: the development of cities mainly relies on the Internet, through which the Internet of Things and the Internet are closely combined to achieve technological innovation and application. Compared with the urban sustainability framework, the modern technology and “intelligence” in the smart city framework have received more attention. Based on the two major hidden dangers of the robo-advisory service platform's regulatory risk control dilemma and investor irrational emotions, this study innovatively proposes a platform governance analysis framework of “platform risk supervision + investor decision-making capabilities” [8]. From the two paths of platform supervision and investor irrational sentiment, build a robo-advisory service platform risk prediction model and an investor's emotional decision-making model for the robo-advisory service platform, so as to conduct targeted governance on the robo-advisor service platform from different perspectives. In addition, this research analyzes theories of financial development, technological innovation, and smart city construction, including the theoretical basis of financial development, technological innovation, and smart city construction [9–11], as well as the analysis of the mechanism of action among financial development, technological innovation, and smart city construction.

## 2. Fintech Platform Risk Assessment Regulation Algorithm Method

### 2.1. The Module Division and Overall Architecture of the Robo-Advisory System

Robo-advisor generally refers to robot financial management. Robot financial management is the introduction of artificial intelligence into traditional financial advisory services, instead of physical robots helping customers manage financial affairs. Instead, it provides automated investment portfolio recommendations through computer program algorithms based on the investment objectives and risk tolerance set by the demander through online interactions. Unlike traditional counter-counter face-to-face financial management services, which require many service personnel, the purpose is to improve efficiency. The robo-advisor is divided into four major functional modules, as shown in Figure 1. The first functional module is the data collection module, which is responsible for the collection of Exchange Traded Fund (ETF) transaction data and the calculation of the recent rate of return [12]. The data flow from the information collection layer, and its main function is to collect analysis data related to the assessment object and the information technology risk, including assessment task information, basic information of banking business system, bank information technology management, business process status investigation, as well as vulnerability threats and asset value identification based on business system assets. ETF mainly involves three participating entities, namely promoters, trustees, and investors. The promoters and fund product founders are generally stock exchanges, large fund management companies, and securities companies. The trustee is entrusted by the promoter to custody and control all the assets of the stock trust portfolio. Since the index ETF adopts an indexed investment strategy, unless the index changes, the trustee generally does not need to adjust the stock portfolio from time to time, but the trustee of the management investment company ETF has a certain degree of freedom of investment decision-making power. Trustees are generally financial institutions such as banks, trust, and investment companies. The second functional module is the user management module, which is responsible for the management of user accounts, the management of user risk tolerance ratings, and the management of user investment portfolios. The third functional module is the portfolio recommendation module, which is responsible for the preprocessing of transaction data, the calculation of the recommended portfolio (completed through the portfolio model), and the storage of the recommended portfolio. The fourth functional module is the monitoring and rebalancing module, which is responsible for simulating the value trend of the investment portfolio, monitoring the deviation of the portfolio fund allocation ratio during the calculation of the trend, and adjusting the ratio back to the recommended state when the deviation exceeds the threshold.

The article studied the supervision of robo-advisors, but as far as the existing robo-advisors papers are concerned, more research focuses on the fields of finance and information engineering. Therefore, in the writing process, the research results of robo-advisors in economics, finance, and other related disciplines are integrated, starting from law or economic law, and understanding robo-advisors from as many angles and dimensions as possible.

The main logic processing and calculation work in robo-advisors are concentrated on the server, and the front-end is mainly responsible for sending requests and processing a small amount of data, which are a typical application type suitable for B/S architecture [13–15]. Based on this, the entire system is divided into three parts: data storage, server, and Web front-end. The overall system architecture is shown in Figure 2. Among them, the data storage part is responsible for storing user information, historical ETF transaction data, the recent daily rate of return of each ETF, and information about recommended investment portfolios and user investment portfolios. The server is responsible for receiving front-end requests, performing logical processing, reading and writing data, and sending responses to the front-end. The web front-end is responsible for providing users with operating interfaces, sending requests to the server, and receiving and displaying the results returned by the server to users.

### 2.2. Adaptation Module Design

Intelligent analysis is divided into user analysis and investment analysis. User analysis is to analyze according to the evaluation questionnaire filled by the user during the user data acquisition stage, to classify different customers, and to allocate the proportion of large-scale assets according to the results of the rating.

When securities companies develop robo-advisor projects, they collect the “views” of retail customers through the analysis of retail customer historical data, market peer experience, and massive transaction data mining, complete the establishment of customer characteristic factors, and analyze and summarize the customer characteristic factor library. And through the subdivision of factors, it can be summarized into categories such as customer's overall characteristics, transaction characteristics, investment style, investment strategy, investment skills, and position status, including multiple characteristic factors. The process of collecting customer characteristic factors is shown in Figure 3.

At the same time of user analysis, investment analysis is also carried out. Investment analysis is based on the analysis of fund data obtained in the data acquisition stage. Investment analysis is divided into two steps. The first step is to select the investment target. When selecting the target, it can first determine the broad categories of assets, and select several outstanding funds of various assets to join the asset pool through data analysis. The specific choice can be based on fund company ranking, fund manager ranking, fund performance ranking, and some fund evaluation indicators, such as Sharpe ratio and maximum retracement of the interval, through these methods to select the best funds. A comprehensive analysis of the customer's historical investment characteristics and investment skills will be carried out, and the customer's trading operations will be recorded in the customer's characteristic factor system, and the investment characteristic factors of the company's investment consultants will also be collected [16]. The characteristic factors of the two include industry selection, individual stock selection, profit and loss ratio, high-frequency trading period, timely stop loss rate, timely profit settlement ability, risk control ability, industry preference, position control, individual stock preference, and other characteristic vectors. Using the similar formula calculation method in big data, the vector distance between the customer and the investment adviser is calculated, and the distance represents the similarity between the two. The size of the distance and the level of similarity are positively correlated, that is, the closer the distance, the higher the similarity between the two. For comparison, the system will focus on recommending top five investment advisors with matching degrees to customers, showing their views, simulated investment portfolios, investment advisory products, and self-selected stocks. In strict accordance with the relevant measures for the management of industry investment advisors, investment advisors can provide clients with securities advisory services and investment advisory portfolio products.

The calculation method of matrix element *D*(*i*, *j*) in the similar formula calculation method in big data is as follows:

(1) $$\begin{array}{c} D\left(i,j\right)=d\left(i,j\right)+\min\left\{D\left(i-1,j\right),D\left(i,j-1\right)\right\}, \end{array}$$

where *d*(*i*, *j*) represents the distance between the *i*-th point in the sequence *X* and the *j*-th point in the sequence *Y*.

For the similarity distance of two time series:

(2) $$\begin{array}{c} \Delta \;D=\min\left\{D\left(i-1,j-1\right),D\left(i,j-1\right),D\left(i-1,j\right)\right\},\\ D{\left(i,j\right)}_{\beta }=d\left(i,j\right)+\Delta \;D. \end{array}$$

In addition, the stock market is very time-sensitive. Most of the research on the historical trend of stocks is to have a better prediction of the future. It is hoped that similar stocks will have similar trends in the future. Although the future trend of stocks cannot be fully estimated, it is possible to make appropriate guesses from recent information dynamics. Therefore, the more similar the two stock sequences are in the later time, it means that the two time series are more similar. Therefore, this research improves the similarity calculation method, introduces exponential weighted moving average, enhances the similarity of recent patterns, and weakens the similarity weight far away from the current time. The weighted formula is as follows:

(3) $$\begin{array}{c} D\left(i,j\right)=\beta \left(i,j\right)+\left(1-\chi \right)\min\left\{D\left(i-1,j\right),D\left(i,j-1\right)\right\}, \end{array}$$

where *β* is the weight coefficient.

The formula for attractiveness is as follows:

(4) $$\begin{array}{c} X\left(m,n\right)=s\left(m,n\right)-\max\left\{a\left(i,k\right)+s\left(i,k\right)\right\}, \end{array}$$

where (*m*, *n*) is the similarity between points *m*, *n*.

In the iterative update, similar clustering of big data may oscillate due to some noise data, so the smoothing factor *α* is introduced for control, which is also called the damping coefficient, and the previous trend is considered in the current trend direction. The formula for one iteration of attraction *X* and belonging *A* is as follows:

(5) $$\begin{array}{c} X=\left(1-\alpha \right)X_{T-1}+\left(1-\lambda \right)X_{T-1},\\ A=\left(1-\alpha \right)A_{T-1}+\left(1-\lambda \right)A_{T-1}. \end{array}$$

The similarities between stocks are described in different ways, and then the stocks are divided into categories by splicing different clustering algorithms. Exploring the pros and cons of the similarity of different methods for stock time series data, and the differences between different clustering algorithms, select the most suitable clustering algorithm for stock classification, and enhance the accuracy of stock classification.

In Markowitz's modern portfolio theory, indicators to measure returns and risks are proposed:

(6) $$\begin{array}{c} R=\sum_{i=1}^{n}wr, \end{array}$$

*R* is the expected return of the asset portfolio.

The formula for portfolio risk is as follows:

(7) $$\begin{array}{c} \lambda^{2}=\sum_{i=1}^{n}\sum_{j=1}^{n}w_{i}w_{j}\lambda_{ij}. \end{array}$$

Establishing an effective investment portfolio by finding the minimum portfolio standard deviation under the condition of a given expected return *R*:

(8) $$\begin{array}{c} \text{min}\lambda^{2}=\sum_{i=1}^{n}\sum_{j=1}^{n}w_{i}w_{j}\lambda_{ij}+\gamma ,\\ \text{STR}=\sum_{i=1}^{n}w_{i}r_{j}. \end{array}$$

Using the risk parity model to optimize the combination formula is as follows:

(9) $$\begin{array}{c} \min f=\sum_{i=1}^{n}\sum_{j=1}^{n}{\left[w{\left(\Omega w\right)}_{i}-w{\left(\Omega w\right)}_{j}\right]}^{2}. \end{array}$$

The formula for calculating the consistency CI is as follows:

(10) $$\begin{array}{c} \text{CI}=\frac{\left(\lambda -N\right)}{\left(N-1\right)},\\ \text{RI}=\frac{\left(K-N\right)}{\left(N-1\right)}. \end{array}$$

where *N* is the order of the judgment matrix.

Calculation consistency CR:

(11) $$\begin{array}{c} \text{CR}=\frac{\text{CI}}{\text{RI}}. \end{array}$$

### 2.3. Portfolio Recommendation Module

Existing investment advisory platforms generally use two methods for user analysis to determine the investment ratio. One is to give a few fixed investment ratios for users to choose, such as the Betterment website. This result is actually more inclined to the user's subjective risk perception and ignores the user's objective conditions. It is very likely that the investment results will not match the customer's own situation. The second method is to divide the product portfolio's effective frontier in equal proportions to match the user's risk level. The result of this is not rigorous, and the difference in the choice of products in the effective frontier will also cause great deviations in the configuration results.

The portfolio recommendation module is the core of the entire robo-advisor. It is responsible for preprocessing the recent returns of each ETF, calculating the recommended portfolio through the portfolio model calculation, and storing the recommended results to disk. The optimized investment portfolio model is adopted in the implementation. The preprocessing of the recent returns of each ETF, including the processing of missing data items, and the calculation of the mean and covariance matrix of the returns based on the data. First, take the JSON string of the recent return rate of each ETF from the MongoDB collection return-recent and convert it to the Data Frame type in the memory to obtain the return rate of 82 ETFs in the last 200 trading days. If there are missing items, it means that the corresponding single ETF stopped trading on the trading day due to some reasons of its own. Therefore, the return rate of the day is 0, and 0 can be directly added to the missing items. After dealing with the missing items in the data, it is necessary to calculate the mean return rate and the covariance matrix. Using Pandas to realize the EWM method to calculate the statistical characteristics of the mean and variance of the rate of return, and then use them as the input of the portfolio model, and run the model to get the recommended portfolio. The calculation of the portfolio model takes a lot of time, and it takes several hours in the serial case. The model needs to calculate the number of ETFs contained in the portfolio *K* = 6,7,8,9,10, respectively. Therefore, parallel operation can be realized for different *K* values. Because of the existence of the global interpreter lock in the Python language, only one thread can execute at any time, so the parallel implementation based on the multiprocess is adopted in the implementation, and the running time of the parallel implementation of the portfolio model has dropped to about half an hour.

There is a certain correlation between financial development and technological innovation:

(12) $$\begin{array}{c} \text{LNP}=C+\lambda_{1}\text{SCID}+\lambda_{2}\text{GS}+\lambda_{3}\text{LNF}, \end{array}$$

SCID is the smart city development index.

The dynamic panel model is as follows:

(13) $$\begin{array}{c} {\text{SDI}}_{\text{IT}}=\lambda_{1}\text{SDI}+\lambda_{2}{\text{SDI}}_{2}+\lambda_{3}\text{Lnp}+\lambda_{4}\text{Finance}+\lambda_{5}\text{Control},\\ \text{SDI}=\lambda_{1}\text{LNP}+\lambda_{2}\text{Control}+\gamma . \end{array}$$

Among them, SDI and SDI_2_ represent the SDI index lagging one and two periods, respectively.

### 2.4. Database Implementation

The database of this evaluation system uses SQL-Server. In the implementation process, in order to facilitate the replacement of other database software in the future, this system uses SQL standard statements instead of calling SQL-Server specific functions. Designing a database is to classify tables according to dictionary tables and data tables. Among them, the dictionary table is used to define the data used in the coding. These data have been defined as rules at the beginning of the evaluation, such as asset importance assignment table, fragile assignment table, and asset type, and basically, no addition, deletion, and modification operations are performed. Data tables are often added and deleted during the evaluation process, such as asset identification tables, business system tables, and risk management tables. The asset value assignment information is shown in Table 1.

### 2.5. The Design of the Display Module of the Robo-Advisor System

The robo-advisory system displays a “360-degree stereo view” of customers. The comprehensive investment ability of customers is scored through multiple dimensions such as risk control ability, investment ability, ability to grasp opportunities, and operation ability, and the score is compared with the average score of stock customers to form a “customer profile,” and fully mine customer transaction data to obtain customer investment habitual preference factors. Opening the page of the robo-advisor system to display the timing ability and risk control ability of the customer's investment ability analysis, and display the score and the average score of securities customers. It also displays customer characteristics obtained through testing: turnover rate, preferred industry, relevance of investment and research reports, preferred investment products, preferred risk, degree of concentration or divergence of holdings, and long, medium, or short-term investment risks, etc. Asset risk information is shown in Table 2.

After the investment advisory system configures the investment ratio, feedback is required. The result of the investment portfolio analyzed by the intelligent algorithm is fed back to the customer. The content includes the expected return rate, return volatility, investment asset types and their allocation ratios, and investment recommendations. The investment proposal states the basis of the investment portfolio and the customer's risk tolerance. Customers can invest according to investment recommendations.

Regarding how to recommend suitable financial products to suitable customers, it is assumed that the influence conditions of customers choosing to purchase financial products are customer investment experience, risk level, capital turnover rate, capital scale, expected rate of return, subscription threshold, investment cycle, and investment strategy. Through the simulation system, the purchase rate of different financial products, the order in which customers with the same capital scale purchase products and the product category with the highest purchase probability for customers with the same risk level are calculated. The intelligent model self-learns, trains, and tests the model to construct the most suitable model scheme. At the same time, the weight adjustment of subjective weighting method and the screening rules of customer suitability conditions are added to form a product recommendation list.

The similarity rate of rise and fall in the same category refers to the probability that stocks in the same category will rise and fall in the same direction for a period of time in the future. This article uses SDI to represent the same direction similarity rate of rise and fall, and its calculation method is as follows:

(14) $$\begin{array}{c} \text{SDI}=\frac{\sum_{i}^{N}\max\left\{I_{1},I_{2}\right\}/m}{N}. \end{array}$$

Among them, *N* is the number of categories.

The similarity rate of rise and fall in the same direction *Z*_*D*_ is as follows:

(15) $$\begin{array}{c} Z_{D}=\frac{\alpha *\text{SDI}/\lambda }{\left(\text{PVI}+\beta \right)*\left(\lambda +\beta \right)}=\frac{\alpha *\text{SDI}}{\lambda \left(\text{PVI}+\beta \right)*\left(\lambda +\beta \right)}. \end{array}$$

Let *Q* denote the optimal value of the second-stage problem, which is related to the random parameters and the first-stage decision *X*.

(16) $$\begin{array}{c} Q=\min q\left(y,\xi \right),\\ w\left(y,\xi \right)=h\left(y,\xi \right)-G\left(y,\xi \right). \end{array}$$

Then the stochastic programming model *S*_*G*_ of the compensation problem has the following form:

(17) $$\begin{array}{c} S_{G}=\min f\left(x\right)+E\left(x,\xi \right). \end{array}$$

Nested optimization model:

(18) $$\begin{array}{c} W\left(\xi \right)Z_{1}=H_{1}\left(\xi_{1}\right)-G\left(\xi_{1}\right),\\ W_{T}\left(\xi \right)Z_{T}=H_{T}\left(\xi_{1}\right)-G\left(\xi_{1}\right)Z_{T-1}, \end{array}$$

where *ξ* is a random variable.

## 3. Results of Risk Assessment and Regulation of Financial Technology Platforms

Financial technology companies rely on advanced technology to settle in the market competition, and improper disclosure of internal technical personnel of the company, vulnerabilities in the internal technical system of the company, and improper release of corporate products and services that may all cause the leakage of key corporate technologies. Once the technology is leaked, imitated, or plagiarized by market competitors, what the company loses is not only the waste of the huge investment in research and development in the early stage but also the core competitiveness and potential business opportunities for survival in the market. This blow to enterprise development may be devastating. The main risks of financial enterprises are shown in Figure 4.

Due to various historical reasons, the financial industry will not be linked with “good user experience” and “focus on user needs” in people's vision. On the contrary, it will give people the impression of scarce resources and high service attitude. However, with the impact of the Internet, companies that pay more attention to convenient operation and timely service information will be more favored by users. With the development of Internet finance, according to statistics, it is estimated that in 2021, the number of online payment users will reach approximately 1.33 billion. The payment method statistics are shown in Figure 5. In recent years, the introduction of fast payment in more and more industries shows that the upper limit of the development of smart cities is more far-reaching than people think. Through the introduction of technical means, the convenience of urban residents' life has been further improved, and the use of scientific and technological means has given the government more choices in urban governance and prevention.

For the spot silver from January 01, 2017 to June 05, 2017 on the precious metals exchange in City A and the spot silver 9995 on the precious metals trading center in City B, three *K*-line data of 60 min, 180 min,, and 240 min were used, use the similar formula calculation method in calculating big data to test the conventional accuracy of parameters, and simultaneously monitor the resource utilization of the server. Part of the result data is shown in Table 3.

During the test, the tested function of the system did not run abnormally under the system constraints, which affirmed the guiding role of the similar formula calculation model in the big data on the spot real market. Judging from the test results, the algorithm in this study has successfully made a profit for 25376 times in a total of 30564 transactions, and the accuracy rate is as high as 83.04%.

Based on the above, the risk values of the three major risk domains of bank information technology risk are 54.05, 51.63, and 64.28, respectively. The three risk domains are weighted by collecting opinions from multiple parties, and the final weighted risk assessment results are shown in Table 4.

When clustering data, it is necessary to calculate the distance between different time series separately. Usually, when calculating the distance, the base of the series is different, which will cause large errors. These errors sometimes lead to bizarre data results. The similar formula calculation method in big data is used to solve such problems and speed up the calculation. The timing trend before and after standardization is shown in Figure 6.

The higher risk values in the management domain are information security (19%), information system development, testing and maintenance (21%), information technology operation (30%), and business continuity management (30%). The comparison of risk values in the management domain is shown in Figure 7.

Under the management support center, there are departments such as affairs, finance, project management, and the head of the department reports to the head of the management support center. There is no separate compliance department, intellectual property department, risk control department, and internal audit department that directly report to the board of directors. All compliance, intellectual property, risk control, and internal audit functions are currently concentrated in the legal department. The company's main intellectual property rights, personnel status, and financial status in the past three years are shown in Table 5.

Experiments found that a single LSTM and AVG algorithm is difficult to reduce the loss of the model, and under-fitting occurs. Therefore, the LSTM and AVG algorithms cannot effectively explain the investor emotional decision model. Due to the enhanced feature extraction ability of the risk assessment regulation algorithm and the algorithm of this paper, which integrates Attention, it has a better fit to the investor's emotional decision data, the loss continues to decline, and achieves a relatively stable result. Among them, the risk assessment regulation algorithm model in this study makes the final loss smaller. The loss reduction degree of the four algorithms is shown in Figure 8.

The accuracy of various algorithms is shown in Table 6, which shows that the accuracy of the two-way LSTM and the similar formula calculation method in the fusion of big data has been greatly improved on the basis of a single LSTM and AVG network, by 17% and 10%, respectively. Although the similar formula calculation method in big data integrated with Attention has stronger feature extraction capabilities (with an accuracy of 88%), due to the lack of data on the robo-advisory service platform itself, there may be an overfitting problem. Therefore, the experimental results show that the similar formula calculation method in big data can better explain the emotional decision-making ability of the robo-advisor service platform investors, which provide algorithmic support for the subsequent emotional calculation of platform investors.

Based on the similar formula calculation model in the fusion of big data with experimental training, this study uses Python language and Pytorch framework to calculate sentiment scores for the eight major platform reviews, takes the average value, evaluates the ranking, and compares it with the platform's own comprehensive strength ranking. The specific ranking and sentiment score are shown in Figure 9. The experiment found that investors' risk analysis and platform selection capabilities are still insufficient, and investors' emotional decision-making on the robo-advisor service platform has a large gap with the official platform's comprehensive strength. For example, Huitou Bank ranks very high in the official comprehensive strength announcement, but investors are not optimistic about its evaluation, only reaching a score of about 0.2. It is comprehensively found that investors still lack the ability of rational risk identification and platform selection for robo-advisory service platforms. This experiment explores the characteristics of relevant investor comments on the robo-advisory service platform and the concerns and emotional characteristics of investors on the robo-advisory service platform. First, construct a domain dictionary, segment words, remove stop words, and extract keyword frequencies from the cleaned comment data. It can be found that keywords such as “income,” “risk,” “loss,” “handling fee,” and “fund” appear more frequently, which are the main points that investors pay attention to. The statistical results of investors' attention to keywords are shown in Figure 9.

## 4. Discussion

In the era of “AI for all people,” computers, as the basic tools for processing work, can help people deal with various tedious and repetitive tasks, and they also have a place in the field of financial information analysis. By categorizing this information, it is convenient for people to obtain information that is useful to them. The main research content of this subject is to use computer combined with machine learning methods to classify stocks, and on this basis, to dig out the relationship between stocks or categories, so as to better help users to invest. The market environment of perfect competition often stays at the ideal level, and the realistic market economy often shows the characteristics of imperfect competition. Traditional trade theory believes that in the case of monopolistic competition, open trade can not only expand the scale of the market, deepen industry competition, and increase the degree of international specialization of production, but it can also alleviate the distortion of resource allocation caused by monopoly, make the product price and cost lower, benefit consumers, and improve the national income level.

The financial market plays an important role in the development of the country and the national economy. There are many types of financial products in the financial field. Stock is the most important part of securities, and it is one of the most common investment choices in people's daily life. However, stocks have the characteristics of high risk and high return. Therefore, how to avoid risks and obtain returns when investing in stocks has been a topic of more concern in the society in recent years. Therefore, when studying the relationship between stocks, the relationship between stock categories is considered. Investing in stocks of different categories can be more conducive to reducing investment risks, and the relationship between categories is often more beneficial to investment, because the relationship between many stock categories is often more stable and lasting than the relationship between individual stocks, and a stable relationship can better avoid risks in investment.

Platform speculation and investor irrational sentiments are two important causes of platform risks and turbulence in the financial market environment. On the one hand, the robo-advisory service platform must provide investors with efficient and convenient robo-advisory services, and on the other hand, it must also restrain the uncertain speculative behavior in it and prevent the occurrence of tragic phenomena similar to a large number of P2P online loan investment platforms. This also brings challenges to the government and regulatory authorities. When the regulators provide incentives for robo-advisor concepts to enter China, they are also constantly exploring how to prevent and control the risks of bad investment platforms. For example, the current operation of the robo-advisory service platform needs to obtain the qualification certificate of the China Securities Regulatory Commission, but there are still the phenomena of platform speculation, running off or losing assets of investors.

For example, blockchain technology is based on the concept of “decentralized distributed transparent mechanism,” which replaces the one-way linear relationship of “intermediary–customer” and introduces a highly democratic principle of decentralization into the financial market. Under the above background, the limitations of a single regulatory body, a single regulatory means, and a single regulatory model have become more and more obvious. In the context of financial technology, financial regulatory agencies will fall into a long-term trilemma that they can only achieve two of the three goals of seeking clear rules, maintaining market credibility, and encouraging financial innovation. “The drive of the information regulation model to the power of social regulation” provides a new way of thinking for the socialization and diversification of financial technology regulation. Therefore, information regulation can complement administrative regulation to achieve functional advantages, integrate regulatory resources from the government, market and society, and build a multilevel compound model of financial technology regulation.

The change from Internet finance to financial technology means that regulatory activities are becoming more complex and professional. However, with the rapid development of technical means, technology is subtly changing the way and value of information regulation, and it is an inevitable trend to reshape information regulation. In the context of financial technology, the content and structure of information regulation have become more and more complex, and instrumental rationality and value rationality have shown a dualistic and potentially unified contradiction in information regulation. As the current Internet financial market is undergoing a period of fierce changes and strong supervision, and a large number of Internet financial platforms are closed or cleared, the market is in a special period of transition from “Internet finance” to “financial technology.” Investors still lack the ability of robo-advisory service platform selection and risk identification, and there are two key points in its governance: on the one hand, investors' irrational decisions account for a large proportion. Platform operators and the government or the Securities Regulatory Commission can enter from this to cultivate investors' sense of rational investment, including the popularization of relevant financial investment knowledge and attention to important risk characteristics. On the other hand, it is more important to supervise the compliance operation of the platform and restrict its disclosure of relevant characteristic information. For example, investors are concerned about the income, profit and loss, product structure, etc., and review them, which promotes the sound development of robo-advisors in China and builds a benign investment environment for investors.

Monitoring the problems and deficiencies in the financial markets of various regions, by introducing interactive items, helps to examine the degree of financial development's effect on technological innovation, and can discover and evaluate the degree of integration of financial development and technological innovation in various regions, check whether local financial institutions are in place in implementing the state's policy on financial support for innovation and development. On the basis of having a clear understanding of the financial development and technological innovation of various regions, it helps all regions to proceed from the actual situation and in-depth exploration of the specific path and the best way of the integration of technology and finance. Practicing the spirit of the “18th National Congress” promotes the realization of the goal of an innovative country by enhancing the role of finance in technological innovation. With the continuous in-depth research on smart cities, the focus of research is gradually starting from the nature and connotation of urban construction from what is a smart city and how to build a smart city. It not only evaluates the sustainability of urban construction but also pays more attention to the sustainable development of people. With the diversification and standardization of research, smart cities in particular have now developed into a national strategic plan; how to use better methods to construct and how to evaluate the performance of a complex system of smart city financial projects has become a research object that needs to be focused on nowadays.

## 5. Conclusion

Driven by digitization and informatization, financial technology plays an important role in promoting financial decentralization and financial democratization. The use of scientific and technological means and Internet technology to provide convenient and accurate inclusive financial services for long-tail customers has realized the decentralization and multicentralization of power in the financial market. This article's research on Internet financial information regulation is still mainly based on the context of “Internet finance.” The research on the paradigm of information regulation in the context of “financial technology” is still insufficient, and the research on the characteristics of the integration of information regulation and technology needs to be in-depth. In addition, the study of relevant Internet financial judicial cases still needs to be further excavated and sorted out. This study combines the latest developments of robo-advisory products, comprehensively analyzes the actual situation of robo-advisory platforms, and constructs a model of influencing factors about the use behavior of robo-advisors. This study analyzes the investor's emotional decision-making ability based on the information asymmetry theory and the bounded rationality theory of economic behavior. The existing domestic regulatory policies may not be able to effectively supervise robo-advisory service platforms. In such an environment, robo-advisory services are also difficult to meet the needs of investors. One of the important reasons for this is the irrational investment sentiment of investors. At present, investors' investment philosophy is not yet mature; for example, investors generally value short-term returns.

## Figures and Tables

**Figure 1:** Module division of the four major functional modules.

**Figure 2:** Overall system architecture.

**Figure 3:** The process of collecting customer characteristic factors.

**Figure 4:** Main risks of financial companies.

**Figure 5:** Payment method statistics.

**Figure 6:** Time series trends before and after standardization.

**Figure 7:** Comparison of risk values in the management domain.

**Figure 8:** Loss reduction degree of four algorithm learning.

**Figure 9:** Statistics of investors' attention to keywords.

**Table 1:** Asset value assignment information.

Field name	Type of data	Length	Describe
ID	Int	4	Identification number
Name	Nvarchar	25	Asset materiality description
Rate	Int	4	Value of the asset
Description	Nvarchar	230	Description information

**Table 2:** Asset risk information.

Field name	Type of data	Length	Describe
ID	Int	4	Identification number, primary key
Relevance ID	Int	5	The vulnerability threat association table ID is set as a foreign key related to the vulnerability threat association table
Device ID	Int	6	Corresponding to the asset ID in the vulnerability threat association table t_ relevance
Threat ID	Real	4	Corresponding to the vulnerability ID in the vulnerability threat association table t_ relevance

**Table 3:** Part of the result data.

Variety name	Number of successful long signals	The number of successful short signals	Short-selling success rate
1	131	131	0.8771
2	111	13	0.8193
3	101	10	0.8193
4	101	13	0.8713
5	103	107	0.81
6	110	13	0.8783
7	117	11	0.8187
8	107	13	0.8731

**Table 4:** Final weighted risk assessment results.

Risk domain name	Risk domain weight	Risk domain risk value	Risk domain weighted risk value
Management domain	0.3	54.05	10.88
Business process domain	0.3	51.63	15.78
Business system domain	0.5	64.38	33.64

**Table 5:** The company's main intellectual property rights, personnel status, and financial status in the past three years.

Year	Net assets	Sales revenue	Total profit
2019	24172.17	440.21	−2441.41
2018	26611.91	121.47	−2161.49
2017	29777.29	5.67	−10022.72

**Table 6:** Accuracy of various algorithms.

Model/evaluation index	Net assets (%)
AVG	70
Bidirectional LSTM	71
Similar formula calculation method in big data	86
Similar formula calculation method in big data fused with attention	88

## Data Availability

The data that support the findings of this study are available from the corresponding author upon reasonable request.

## References

[1] Yeh J.-Y., Chen C.-H. (2020). A machine learning approach to predict the success of crowdfunding fintech project. *Journal of Enterprise Information Management*.

[2] Menouar H., Guvenc I., Akkaya K., Uluagac A. S., Kadri A., Tuncer A. (2017). UAV-enabled intelligent transportation systems for the smart city: applications and challenges. *IEEE Communications Magazine*.

[3] Bo T., Zhen C., Hefferman G. (2017). Incorporating intelligence in fog computing for big data analysis in smart cities. *IEEE Transactions on Industrial Informatics*.

[4] Brundu F. G., Patti E., Osello A. (2017). IoT software infrastructure for energy management and simulation in smart cities. *IEEE Transactions on Industrial Informatics*.

[5] Mosannenzadeh F., Bisello A., Vaccaro R., D’Alonzo V., Hunter G. W., Vettorato D. (2017). Smart energy city development: a story told by urban planners. *Cities*.

[6] Badii C., Bellini P., Cenni D., Difino A., Nesi P., Paolucci M. (2017). Analysis and assessment of a knowledge based smart city architecture providing service APIs. *Future Generation Computer Systems*.

[7] Daniel C., Mario C., Giovanni P., Cristian D. (2017). A fuzzy-based approach for sensing, coding and transmission configuration of visual sensors in smart city applications. *Sensors*.

[8] Yuan Y.-H., Tsao S.-H., Chyou J.-T., Tsai S.-B. (2020). An empirical study on effects of electronic word-of-mouth and Internet risk avoidance on purchase intention: from the perspective of big data. *Soft Computing*.

[9] Yue H., Liao H., Dong Li, Chen L. (2021). Enterprise financial risk management using information fusion technology and big data mining. *Wireless Communications and Mobile Computing*.

[10] Xu Z., Zhu G., Metawa N., Zhou Q. (2022). Machine learning based customer meta-combination brand equity analysis for marketing behavior evaluation. *Information Processing & Management*.

[11] Gu C. (2022). Application of data mining technology in financial intervention based on data fusion information entropy. *Journal of Sensors*.

[12] Chen Y., Zheng W., Li W., Huang Y. (2021). Large group Activity security risk assessment and risk early warning based on random forest algorithm. *Pattern Recognition Letters*.

[13] Khalaf O. I., Abdulsahib G. M. (2021). Optimized dynamic storage of data (ODSD) in IoT based on blockchain for wireless sensor networks. *Peer-to-Peer Networking and Applications*.

[14] Namasudra S., Roy P. (2018). PpBAC. *Journal of Organizational and End User Computing*.

[15] Zhang Y., Huang H., Yang L.-X., Xiang Y., Li M. (2019). Serious challenges and potential solutions for the industrial Internet of things with edge intelligence. *IEEE Network*.

[16] Al-Momani A. M., Mahmoud M. A., Ahmad M. S. (2018). Factors that influence the acceptance of Internet of things services by customers of telecommunication companies in Jordan. *Journal of Organizational and End User Computing*.

